The article "Exploring the Ferroptosis Mechanism of Zhilong Huoxue Tongyu Capsule for the Treatment of Intracerebral Hemorrhage Based on Network Pharmacology and In Vivo Validation" was published in 2022. Journal: Evid Based Complement Alternat Med.

# Exploring the Ferroptosis Mechanism of Zhilong Huoxue Tongyu Capsule for the Treatment of Intracerebral Hemorrhage Based on Network Pharmacology and *In Vivo* Validation

**DOI:** 10.1155/2022/5033135

**Published:** 2022-09-25

**Authors:** Lixia Wang, Wei Ren, Li Wang, Linshen Mao, Maryam Mazhar, Chen Zhou, Houping Xu, Sijin Yang

**Affiliations:** ^1^Hospital of Chengdu University of Traditional Chinese Medicine, No. 39 Shi-er-qiao Road, Chengdu 610072, China; ^2^National Traditional Chinese Medicine Clinical Research Base of the Affiliated Traditional Chinese Medicine Hospital of Southwest Medical University, No. 182 Chunhui Road, Longmatan District, Luzhou 646000, China; ^3^Institute of Integrated Chinese andWestern Medicine of Southwest Medical University, Luzhou 646000, China; ^4^Preventive Treatment Center of the Affiliated Traditional Chinese Medicine Hospital of Southwest Medical University, Luzhou 646000, China

## Abstract

**Objective:**

The purpose of this study is to explore the mechanism of the Zhilong Huoxue Tongyu (ZL) capsule in the treatment of intracerebral hemorrhage (ICH) via targeting ferroptosis based on network pharmacology.

**Methods:**

The active ingredients and related key targets of the ZL capsule were screened using the Traditional Chinese Medicine Systems Pharmacology Database and Analysis Platform (TCMSP). The gene ontology (GO) enrichment analysis and Kyoto Encyclopedia of Genes and Genomes (KEGG) enrichment analysis were also performed. Finally, identified targets were validated in an *in-vivo* model of ICH.

**Results:**

A total of 30 active ingredients and 33 intersecting targets were identified through a TCMSP database search. Ingredients-Targets-Pathways network was constructed to filter out the key targets according to the degree value. TP53 was selected as the key target. The *in-vivo* validation studies demonstrated that TP53 was down-regulated and GPX4 was upregulated in rats following ZL capsule treatment.

**Conclusions:**

It is concluded that the ZL capsule could alleviate ICH in a muti-target and multi-pathway manner. ZL capsule could alleviate ICH by inhibiting ferroptosis, and TP53 is identified to be the potential target. Further research is needed to clarify the detailed anti-ferroptotic mechanism of the ZL capsule.

## 1. Introduction

Spontaneous intracerebral hemorrhage (ICH) refers to the hemorrhage within the brain parenchyma [1]. It is characterized by high mortality and disability rate with a globally rising prevalence [2]. Recently, the prevalence of ICH in young is increasing, and hypertension is the main cause of ICH in populations of Asia young adults [3], which has imparted a heavy social and economic burden. Although there is a great deal of attention focused on the development of effective treatment for ICH, there is still a lack of available Class I Level A treatment modalities for ICH patients [4]. Currently, the available treatment options for ICH employ supportive care management and/or surgical removal of hematoma [5], both of which are not ideal for significantly ameliorating ICH. Secondary brain injury (SBI) occurs due to neurotoxicity induced by deleterious byproducts of red blood cell lysis, especially free iron, which leads to inflammation, cytotoxicity, and oxidative damage [6, 7], has been critical effectors of neurological deficits after ICH [8]. Therefore, it is meaningful to figure out the mechanisms of SBI to develop an effective target-based treatment for ICH.

Traditional Chinese medicine is a characteristic module of medicine in China with a history of thousands of years. A large number of Chinese herbal medicines have shown neuroprotective effects after ICH. ZL capsule is a patent traditional Chinese medicine consisting of five traditional Chinese medicines: *Huang qi*, *Di long*, *Da xue teng*, *Gui zhi*, and *Shui zhi*, the detailed information was shown in Table 1. Our previous results suggested that the ZL capsule could reduce the volume of intracranial hematoma in patients (*n* = 30) and improves stroke-related scale scores obviously [9]. Additionally, the ZL capsule was able to alleviate ICH injury outcomes such as inflammation, cerebral edema, neuronal apoptosis, and behavioral cognition in animal studies [10–12]. However, the specific mechanism of the ZL capsule for the treatment of ICH remains unknown.

Ferroptosis is an iron-dependent regulated form of cell death caused by the accumulation of lipid-based reactive oxygen species (ROS) [13]. It has been proven that ferroptosis could coexist with other types of programmed cell death (PCD), such as apoptosis and pyroptosis after ICH [14–16]. The inhibition of ferroptosis shows a therapeutic efficacy against ICH [17, 18]. And glutathione peroxidase 4 (GPX4) is a chief regulator to reducing lipid peroxidation in a glutathione (GSH) level-dependent manner and inhibits the subsequent ferroptosis [19]. Many studies have illustrated that the knock-down or inhibition of GPX4 contributes to lipid peroxidation and subsequent ferroptosis [19, 20]. To find whether the ZL capsule could alleviate ICH via ferroptosis, network pharmacology was performed. Network pharmacology has received great attention as an emerging research technology. The holistic concept, syndrome differentiation, and treatment of traditional Chinese medicine conform to the overall systematic characteristics of network pharmacology [21]. Network pharmacology could provide new insight and approaches for the treatment of disease and drug application.

In this study, we tried to find out the potential targets and mechanisms of the ZL capsule for the treatment of ICH via ferroptosis. First, we got the active ingredients of the ZL capsule, then screened the key targets to obtain GO and KEGG pathway enrichment analysis results. Finally, we screened the target to validate the results of network pharmacology. The flowchart of the experimental procedures of this study was shown in Figure 1.

## 2. Materials and Methods

### 2.1. Predicting Active Ingredients and Targets of ZL Capsule

To obtain the active ingredients and targets of the ZL capsule, the Traditional Chinese Medicine Systems Pharmacology Database and Analysis Platform (TCMSP, https://tcmspw.com/tcmsp.php) [22] and the Uniport Protein Database (https://www.uniprot.org/) [23] were used. TCMSP is a database with the composition of herbal entries, which could help reveal the mechanisms of action of traditional Chinese medicine (TCM) and uncover the nature of TCM theory [22]. According to the characteristics of pharmacokinetics ADME (absorption, distribution, metabolism, and excretion), the results retrieved from TCMSP were screened by two indexes: oral bioavailability (OB) ≥30% and drug-likeness (DL) ≥0.18 to screen the effective active ingredients of ZL capsule [24, 25]. The active ingredients of *Shuizhi* and *Dilong* were screened from TCMID (https://47.100.169.139/tcmid/search/), and then screened in SwissADME to filter ingredients with low gastrointestinal (GI) absorption and SwissTargetPrediction [26] to predict the most probable protein targets [27]. In addition, known targets of compounds whose activity was not predicted were added from published articles. After screening, the information on protein targets was standardized in the Uniport Protein Database. Finally, human target proteins of the ZL capsule were obtained after integration.

### 2.2. Screening of Targets for ICH

To obtain the ICH-related genes comprehensively, we searched target genes from the Human Gene Database (GeneCards database, https://www.genecards.org/) with the keywords “Intracerebral Hemorrhage” and “Cerebral Hemorrhage,” and set the species to “*Homo sapiens*.”

### 2.3. Screening of Targets for Ferroptosis

The related targets of ferroptosis were searched from GeneCards and the Online Mendelian Inheritance in Man (OMIM) database (https://www.omim.org), with the keyword “Ferroptosis.”

### 2.4. Protein-Protein Interaction Network Construction

Protein-Protein Interaction (PPI) plays a key role in the pathogenesis of disease, so the modulation of protein-protein complexes has relevant clinical significance [28]. In this part, the target genes of the ZL capsule for the treatment of ICH were imported into the STRING database (https://string-db.org/) [29] to get the PPI network mapping in the analysis mode of “multiple protein” with the species limited to “*Homo sapiens*” mode. After mapping, the “tsv” format file was imported into Cytoscape to build diagrams for data visualization and integration [30]. The network analyzer plug-in in Cytoscape was used for calculating and ranking the topological parameters to screen the target genes.

### 2.5. GO and KEGG Pathway Enrichment Analysis

To elucidate the pathway and mechanism of the ZL capsule for the treatment of ICH, we collected intersectant targets for GO enrichment and KEGG enrichment analysis in Metascape (https://metascape.org/gp/index.html) for further analysis [31]. Metascape combines gene annotation, interactome analysis, functional enrichment, and membership search to leverage over 40 independent knowledgebases within one integrated portal. GO enrichment is a system used to descript the function of gene in different aspects, such as molecular function (MF), cell composition (CC), and biological process (BP). KEGG enrichment could analyze the pathway involved in the genes. The difference was considered to be statistically significant at *P* < 0.01.

### 2.6. Experimental Validation

#### 2.6.1. Animals and Grouping

Eighteen 2-3 months healthy male Sprague Dawley rats (weighing 250 ± 20 g) were purchased from the Animal Experiment Center of Southwest Medical University. Rats were raised in the SPF animal laboratory of Southwest Medical University and adapted for 1 week. The rats were maintained in a controlled humidity and temperature environment with an alternative 12 h light/dark cycle and ad libitum access to water and food. All experiments were approved by the Animal Ethics Committee of Southwest Medical University (NO. 20211111-002). The animals were randomly divided into three experimental groups: [1] Sham, [2] ICH, and [3] ZL capsule groups with six rats in each group.

#### 2.6.2. ICH Model

An autologous blood injection in adult male rats was used to induce the ICH model in this study [32, 33]. After anesthesia with pentobarbital sodium (40 mg/kg), SD rats were secured on a stereotaxic apparatus (Changsha Meyue Biotechnology Co., Ltd, Hunan, China). And the right basal ganglia (1.5 mm anterior and 3.0 mm lateral to bregma) were inserted into a depth of 6 mm with a microsyringe. Next, within 5 min, 100 *μ*l of autologous blood collected from the tail was injected at a rate of 20 *μ*l/min. Sham-operated rats were intracerebrally injected with a needle without blood injection. During the ICH surgical procedure, the temperature, heart rate, and respiratory rate of animals were monitored.

The neurobehavioral scores of the ICH models were evaluated after the rats were awakened, according to the Zea-Longa neurological deficits score [34], to confirm the establishment of the ICH model. The criteria of the Zea-Longa score are listed in Table 2. Rats with a score of 1–3 were included in the study according to the Zea-Longa score.

#### 2.6.3. Behavioral Studies

The rats were assessed at 1, 3, 5, and 7 days after ICH to evaluate the neurobehavioral outcomes according to the Zea-Longa score and Neurological Severity Score (NSS) [35, 36]. The NSS evaluation included the motor, sensory, balance tests, and reflexes [35].

#### 2.6.4. Drug and Dosing

ZL capsules (Zhilong Huoxue Tongyu Capsule) were provided by the Pharmacy Department of Affiliated Traditional Chinese Medicine Hospital of Southwest Medical University. According to our previous studies, the dosage was converted according to the body surface area of rats as 2 g/kg/day [37]. The ZL capsule was administered orally for 7 days to the ZL capsule treatment group. The ICH group animals were administered with the same dose of normal saline by oral gavage for 7 days.

#### 2.6.5. Quantitative Real Time PCR

The total RNA was extracted by Trizol reagent (TIANGEN, DP419). Reverse transcription was performed using HiFi-MMLV cDNA Kit (Cwbio, CW0744M) to synthesize the cDNA template. PCR primers used for PCR amplification were obtained from Sangon Biotech (Chengdu, China). Quantitative real-time PCR was performed using SYBR Green Kit (Cwbio, CW2601H) in LightCycler 480 (Roche). The reaction program contained 40 cycles of denaturation at 95°C for 15 s and annealing at 60°C for 1 min. The RNA expression levels were calculated by the 2^−ΔΔCt(Quantitation−ComparativeCT)^ method based on the normalization of GAPDH values. The primer sequences used in our study are as follows: TP53: Forward primer: 5′-AGTGGGAATCTTCTGGGACG-3′, Reverse primer: 5′-TCTTTTGCTGGGGAGAGGAG-3′; GAPDH: Forward primer: 5′-CAAGGCTGAGAATGGGAAGC-3′, Reverse primer: 5′- GAAGACGCCAGTAGACTCCA-3′.

#### 2.6.6. Western Blot Analysis

After 7 days of ICH modeling, the cortical brain tissues of each group were collected. The protein expression was extracted via RIPA buffer (Beyotime, Shanghai, China) and the concentrations of protein were measured by a BCA assay kit (Beyotime, Shanghai, China). Protein (48 *μ*g/lane) was separated by 10% SDS polyacrylamide gel at 80 V for 20 min and then 100 V for 1 h, and then transferred onto PVDF membranes (Millipore, Darmstadt, Germany). The membranes were then blocked in 5% BSA (Solarbio, Beijing, China) for 1 h at room temperature. Next, the blocked membranes were incubated with primary antibody anti-TP53 (dilution, 1 : 2,000; Affinity, Jiangsu, China), anti-GPX4 (dilution, 1 : 5,000; Abcam, Cambridge, MA, United States), and GAPDH (dilution, 1 : 5,000; Beyotime, Shanghai, China) overnight at 4°C. The membranes were then washed with TBST and incubated with horseradish peroxidase (HRP)-conjugated secondary antibody (dilution, 1 : 5,000; goat anti-rabbit; Beyotime, Shanghai, China) for 2 h at room temperature. The protein bands were visualized via enhanced chemiluminescence (ECL) kit (Beyotime, Shanghai, China), and the relative protein quantity was determined using ImageJ software (National Institutes of Health, USA).

### 2.7. Statistical Analysis

All data were presented as mean ± standard deviation (SD) and analyzed with SPSS 24.0 software. One-way ANOVA was used to analyze data obtained from multiple groups. *P* value < 0.05 was considered statistically significant.

## 3. Results

### 3.1. Active Ingredients of ZL Capsule

The total ingredients of the ZL capsule were searched through TCMSP and TCMID databases. The detailed information is outlined in Table 3. Based on integrated results of the two databases, *Da xue teng* included 4 active ingredients, 17 in *Huangqi*, 6 in *Guizhi*, 1 in *Shuizhi* and 4 in *Dilong.* It was found that Sargentodoxa cuneate and Cinnamomum cassia Presl contain two similar ingredients (A&B in Table 3). After removing the duplicates, a total of 30 non-repeating ingredients were retrieved.

### 3.2. Target Retrieval and Analysis

Based on identified active ingredients, we further searched the related potential targets. A total of 1351 targets were retrieved, and all the targets' names were standardized in the Uniport Protein Database [20]. After eliminating the duplicate targets, 539 targets remained (Figure 2(c)). Next, we searched ICH-related targets in Genecards database using the keywords, “Intracerebral Hemorrhage” and “Cerebral Hemorrhage,” and we obtained 5379 targets for ICH. After eliminating the duplicate targets, 4338 targets remained. Moreover, we searched the targets of ferroptosis in the Genecards and OMIM database, which displayed 408 ferroptosis-related non-redundant targets.

In order to screen out the target genes of the ZL capsule for ICH, we intersected the targets of the ZL capsule with that of ICH, and a total of 300 overlapping target genes were searched. The related target genes between ICH and ferroptosis were intersected, and 249 target genes were selected. The related target genes between ferroptosis and ZL capsule were intersected, and 40 target genes were selected. To further explore the mechanism of the ZL capsule through ferroptosis in the treatment of ICH, we intersected the intersectant target again and got 33 key target genes. The intersectant targets can be seen in Figure 2(a) and supplementary materials.

### 3.3. PPI Network for the Targets of ZL Capsule

In order to analyze the function between known protein and predicted protein, we conducted a PPI network analysis in the STRING database. More than 33 key genes were imported into STRING, with specie selection as “*Homo sapiens*.” According to the results of STRING, 33 nodes, 180 edges, and 10.9 average node degrees were identified. The results were then imported into Cytoscape in the form of “tsv” to construct the figure of the PPI network. The analysis for the rank of the genes according to the value of degree was performed via network Analyzer tool in Cytoscape. As shown in Figure 2(b), the size of each circular node represented the importance of each gene. The bigger size the of the node, the higher the corresponding degree value. According to the degree value, top 10 genes that were found to be influential targets in the treatment of ZL capsule via ferroptosis are as follows: TP53 [25], TNF [23], EGFR [22], PTEN [22], MYC [21], JUN [21], PTGS2 [18], RELA [16], HMOX1 [15] and GSK3B [15].

### 3.4. GO Enrichment and KEGG Analysis

To investigate the molecular mechanism of the ZL capsule through ferroptosis, GO enrichment and KEGG pathway analysis were carried out on the 33 key genes in the Metascape database. The GO analysis described the function of key targets from three aspects: biological process (BP), cellular component (CC), and molecular function (MF). The detailed results of the GO enrichment analysis were outlined in Figure 3(a). The results indicated that the biological processes of the target ZL capsule for the treatment of ICH via ferroptosis mainly included the response to an inorganic substance (GO: 0010035), response to xenobiotic stimulus (GO: 0009410), regulation of apoptotic signaling pathway (GO: 2001233), negative regulation of phosphate metabolic process (GO: 0045936), gland development (GO: 0048732) and cellular response to organonitrogen compound (GO: 0071417). The enriched molecular functional ontologies mainly included ubiquitin protein ligase binding (GO: 0031625), DNA-binding transcription factor binding (GO: 0140297), kinase binding (GO: 0019900), oxidoreductase activity (GO: 0016491), cadherin binding (GO: 0045296), and phosphoprotein binding (GO: 0051219). The cellular component analysis showed that cell body (GO: 0044297), membrane raft (GO: 0045121), focal adhesion (GO: 0005925), transcription regulator complex (GO: 0005667), vesicle lumen (GO: 0031983), and PML body (GO: 0016605).

Moreover, the KEGG pathway was analyzed for the 33 key genes, as displayed in Figure 3(c) and Table 4. The identified influential pathways include pathways in cancer (hsa05200), hepatitis B (hsa05161), human cytomegalovirus infection (hsa05163), IL-17 signaling pathway (hsa04657), fluid shear stress and atherosclerosis (hsa05418), chemical carcinogenesis—reactive oxygen species (hsa05208), and ferroptosis (hsa04216).

### 3.5. Pathway Network of ZL Capsule Active Ingredients for ICH Treatment Targets via Ferroptosis

In order to figure out the key targets and compounds, Cytoscape was performed to build the ZL capsule active ingredients- ICH key targets-top 11 Pathway network diagram, and the analysis results were arranged, as shown in Figure 3(b), Tables 5 and 6. The degree value of quercetin was found to be 18, Betweenness Centrality was 0.23778696, and Closeness Centrality was 0.51239669. It was indicated that quercetin was the main active ingredient in the ZL capsule for the treatment of ICH. Further, the degree value of crocetin was found to be 6, Betweenness Centrality was 0.08568377, and Closeness Centrality was 0.41059603. For kaempferol, the degree value was 6, Betweenness Centrality was 0.01941172, and Closeness Centrality was 0.41059603. In addition to gene targets, the degree value of PTGS2 was 24, Betweenness Centrality was 0.44995211, and Closeness Centrality was 0.55357143. It was suggested that PTGS2 serve as the major target in the ZL capsule for ICH. For RELA, the degree value was 10, Betweenness Centrality was 0.04458046, and Closeness Centrality was 0.41891892. Similarly, the degree value of JUN was 9, Betweenness Centrality was 0.03443671, and Closeness Centrality was 0.41333333. The degree value of TP53 was 8, Betweenness Centrality was 0.068708, and Closeness Centrality was 0.43055556. Taking together the above three parameters, PTGS2 and TP53 were identified to be the major targets.

Based on our results and previous researchstudies regarding the mechanism of ferroptosis, we selected TP53 as the final target of validation. As the core target in ferroptosis, we further proved that GPX4 participates in the treatment of ZL capsules for ICH via ferroptosis.

### 3.6. Expression Levels of Key Targets in the Treatment of ZL Capsule for ICH in Rats

#### 3.6.1. The Results of Behavioral Tests after ICH in Rats

ICH-induced neurological deficits in rats were assessed by Zea-Longa score and NSS. The Zea-Longa score of the ICH model was significantly increased as compared to the Sham group (*P* < 0.05, Figure 4(b)), but ZL capsule-treated rats had shown decreased score (*P* < 0.05, Figure 4(b)), indicating the ameliorating effect of ZL capsule on neurological damage after ICH. Moreover, the NSS in ICH group was dramatically increased as compared to the Sham group (*P* < 0.05, Figure 4(a)), and the treatment with ZL capsules in ICH rats decreased the NSS level (*P* < 0.05, Figure 4(a)).

#### 3.6.2. Real-Time Quantitative PCR of TP53

The results of mRNA expression levels of TP53 were displayed in Figure 4. Compared with the Sham group, the mRNA expression level of TP53 in the ICH group was significantly increased (*P* < 0.05, Figure 4(c)), whereas, the ZL capsule group showed a dramatically decreased expression level of TP53 (*P* < 0.05, Figure 4(c)).

#### 3.6.3. Western Blot of TP53 and GPX4

For the multifaceted verification, the western blot was performed to investigate the protein expression of TP53 and GPX4, and the results are shown in Figure 4(d). In the ICH group, the TP53 protein expression was upregulated as compared to the Sham group, however, the ZL capsule treatment group demonstrated a significantly decreased protein expression level of TP53 (*P* < 0.05, Figure 4(f)). Moreover, the expression level of GPX4 was significantly decreased in the ICH group as compared to the Sham group, whereas, upregulated in the ZL capsule treatment group (*P* < 0.05, Figure 4(e)).

## 4. Discussion

The SBI after ICH is complicated and multifactorial [8], the key factors that accelerate SBI included hemin, hemoglobin, iron and thrombin, which lead to the occurrence of neuroinflammation, oxidative stress and neuronal death after ICH [38]. And iron deposition could contribute to oxidative stress and lipid peroxidation via Fenton reaction and subsequent ferroptosis [39]. It has been proven that iron overload and accumulation of lipid peroxides and ROS are the basic biochemical characteristics of ferroptosis [40], which has been confirmed to be involved in the onset and development of ICH. Therefore, the occurrence of ferroptosis is closely related to the SBI after ICH. In this study, we attempt to identify the mechanism of the ZL capsule against ICH via ferroptosis with the combination of a network pharmacology approach and experimental validation. And there are 30 active ingredients in the ZL capsule and 539 related gene targets. After topology analysis, quercetin, crocetin, kaempferol, beta-sitosterol, formononetin and isorhamnetin were the important active ingredients found in the ZL capsule for the treatment of ICH. The corresponding gene targets identified include TP53, PTGS2, TNF, JUN etc., which were found to be involved in BP, MF, CC and pathway enrichment. The main pathways included ferroptosis, IL-17 signaling pathway and VEGF signaling pathway. Further experimental verification suggested that the ZL capsule engages ferroptosis inhibition via regulating TP53 for the treatment of ICH.

ZL capsule is a patent traditional Chinese medicine that is composed under the medication rule of *Xuan Fu* theory and Feng medicine, and the clinical application of the ZL capsule has been widely accepted. A systematic review and meta-analysis of the ZL capsule in the treatment of acute cerebral infarction (ACI) suggested that the ZL capsule could ameliorate short-term outcomes of ischemic stroke [41]. Moreover, studies have shown that for treating cerebrovascular diseases, the multi-components of the ZL capsule exert their action via multi-targets of anti-inflammatory, anti-apoptosis, and pro-angiogenesis pathways [9]. Previous studies have reported the coexistence of ferroptosis, autophagy and necrosis in mouse brain tissues after ICH [16], and the inhibition of ferroptosis contribute significantly to the alleviation of neurological outcomes post-ICH [42]. So, it is meaningful to figure out the role of the ZL capsule in the treatment of ICH.

The main mechanisms of ferroptosis include lipid peroxidation, the antioxidant system and iron metabolism after ICH [14]. In our studies, ZL capsules have shown a neuroprotective effect after ICH in rats. It is significant to determine whether ZL capsules could alleviate ICH by modulating the mechanism of ferroptosis. The occurrence and onset of ferroptosis are closely related to oxidative stress [43], therefore the ability of anti-oxidant is important for the inhibition of ferroptosis. Regarding the effective ingredients of the ZL capsule, quercetin is a naturally occurring flavonoid and popularly known as a nutritional anti-oxidant. It has been verified that quercetin is involved in the protection against ICH through suppressing oxidant activity, inflammatory response, and apoptosis [44, 45]. Crocetin is derived from *Crocus sativus* stigmas and has shown antioxidation and neuronal protection in many studies [46]. Trans-crocin 4 (TC4), which quickly hydrolyzes to crocetin after oral administration, can penetrate the BBB without hydrolysis, further mechanism needs to be explored [47]. Kaempferol is a natural flavonoid in plants, with anti-oxidant, anticancer, and anti-inflammatory properties in treating cardiovascular diseases, neurodegenerative diseases, and cerebral ischemic reperfusion injury [48, 49]. Importantly, it has been confirmed that kaempferol ameliorated ferroptosis in ODG/R via Nrf2/SLC7A11/GPX4 axis [50]. From our findings, we can conclude that the active ingredients of the ZL capsule could inhibit ferroptosis after ICH via attenuating oxidative stress.

TP53 is a tumor suppressor protein and is involved in the cellular response to stresses, including hypoxia, DNA damage, and oncogene activation [51]. Previous results suggest that TP53 could regulate ferroptosis in a bidirectional manner. On the one hand, TP53 contributes to ferroptosis via inhibiting SLC7A11 expression or promoting SAT1 and GLS2 expression. On the other hand, TP53 could also suppress ferroptosis through the inhibition of DPP4 activity [51]. At the genetic level, the human Tp53 Arg72Pro (arginine-to-proline amino-acidic substitution) single-nucleotide polymorphism determines neovascularization, brain repair and neurological recovery after ICH, which indicates that TP53 is a therapeutic target in ICH [52]. Further research has shown that the upstream signaling miR-122-5p protects neurons from ICH-induced ferroptosis via miR-122-5p/TP53/SLC7A11 pathway [53]. TP53 is a tumor inhibitor involved in controlling cell survival and division under various pressures [54], such as the metabolism of lipids [55], polyamines [56], iron, and ROS production [57]. Interestingly, many studies have found that TP53 can influence the redox state, thereby modifying the metabolic processes of cells [58] and promoting ferroptosis in oxidative stress conditions [59]. In view of these studies, TP53 is an important regulator for ferroptosis after ICH. Our results have shown that the ZL capsule could downregulate the expression of TP53 and inhibit subsequent ferroptosis after ICH. In order to explain the role of TP53 between ferroptosis and oxidative stress after ICH, further studies are needed.

To sum up, network pharmacology was used in this study, and further validation experiments to explore the potential mechanism of the ZL capsule for the treatment of ICH via ferroptosis were performed. Finally, network pharmacology analyzed that the ZL capsule could alleviate ICH via a multi-target and multi-pathway manner, the results of validation experiments have shown that the ZL capsule could ameliorate ICH via inhibiting ferroptosis through regulating TP53, but more efforts are needed to figure out further mechanism about TP53 and ferroptosis after ICH.

## 5. Conclusion

In this study, we have proven the protective effect of ZL capsules after ICH in rats with the application of network pharmacology and validation experiments. And the active ingredients of the ZL capsule may attenuate oxidative stress after ICH, and further inhibit ferroptosis by modulating the TP53 signaling pathway. These results could support the clinic application of ZL capsules and provide a new sight for the research of ZL capsules and other herbal medicines.

## Figures and Tables

**Figure 1:** Flowchart of the experimental procedures of network pharmacology for the treatment of ZL capsule in ICH via ferroptosis.

**Figure 2:** (a) Venn diagram of 33 intersecting targets among ZL capsule, ICH and ferroptosis. Green represents the 249 intersecting targets between ICH and ferroptosis, blue represents the 40 intersecting targets between ZL capsule and ferroptosis, red represents the 300 intersecting targets between ZL capsule and ICH. The overlapping area reprents 33 intersecting targets among them. (b) The 33 intersecting targets of PPI network diagram among ZL capsule, ICH and ferroptosis. The size of circulars represents the importance of related gene target according to the degree value. The larger circular size, the more important the pathway is. The thicker the line between two targets, the closer the relationship between the two targets is. (c) The active ingredients-targets diagram of ZL capsule. Diamond reprents gene targets, triangle represents related TCM, circular reprents active ingredients, and the same color of circulars mean they are from the same TCM. Additionally, A & B are re-duplicate ingredients between Guizhi and Daxueteng, so we list them separately.

**Figure 3:** (a) The BP, CC and MF enrichment score in GO enrichment analysis of ZL capsule. (b) The ZL capsule active ingredients- ICH key targets- Top 11 pathway network diagram. Different shapes represent different nodes. The circle is the active ingredients, the inverted triangle is the top 11 pathway, and the diamond is the gene target. The node size represents its degree value. The larger the size, the more important the node is. (c) The bubble diagram of top 11 pathway in KEGG enrichment of ZL capsule. The size and color of circulars represent the importance of related pathway. The larger the circular size and the redder the color, the more important the pathway is.

**Figure 4:** (a) NSS score at 1, 3, 5, 7 days after ICH in rats. (^*∗*^*P* < 0.05 between Sham group and ICH group, ^#^*P* < 0.05 between ICH group and ZL capsule group). (b) Zea-Longa score at 1, 3, 5, 7 days after ICH in rats. ^*∗*^*P* < 0.05 between Sham group and ICH group, ^#^*P* < 0.05 between ICH group and ZL capsule group). (c) The mRNA expression of TP53 in cortex of rats after ICH in different groups, *n* = 4 per group. (^*∗*^*P* < 0.05 compared with ICH group). (d) Western blot detection of the expression of TP53 and GPX4 in cortex of rats after ICH in different groups, *n* = 3 per group. (e, f) The relative expression data of TP53 and GPX4 in cortex of ICH rats in different groups (^*∗*^*P* < 0.05 compared with ICH group).

**Table 1:** The name, compatibility and efficacy of five traditional Chinese medicine used in ZL capsule.

Drugs	TCM name	ID	Compatibility of TCM	Efficacy
*Astragalus* membranaceus	Huang qi	HQ	Monarch drug	Strengthening qi, dispelling pathogenic wind, warming yang to promote blood circulation
Pheretima aspergillum	Di long	DL	Minister drug	Feng medicine, eliminating and removing blood stasis, resolving static blood to promote blood circulation
Whitmania pigra whitman	Shui zhi	SZ	Minister drug	Feng medicine, eliminating and removing blood stasis, resolving static blood to promote blood circulation
Sargentodoxa cuneate	Da xue teng	DXT	Minister drug	Dispelling pathogenic wind, promoting blood circulation for removing obstruction in collaterals
Cinnamomum cassia presl	Gui zhi	GZ	Assistant drug	Warming channel and activating blood circulation, reinforcing yang to promote qi

**Table 2:** Zea-longa score.

Zea-longa score	Behavioural performance
0	The rats' behavior without any symptoms of neurological deficit (normal).
1	The rats have dysfunction in stretching the left forelimb (mild neurological deficit).
2	The rats walk in circles and cannot go straight (moderate neurological deficit).
3	The rats lean to the opposite side when standing or crawling (severe neurological deficit).
4	The rats lost conscious and unable to walk.

**Table 3:** The Mol ID, OB and DL of 30 active ingredients in TCMSP database.

ID	Mol ID	Molecule name	OB (%)	DL
DXT2	MOL000096	(−)-Catechin	49.68	0.24
A	MOL000358	Beta-sitosterol	36.91	0.75
B	MOL000359	Sitosterol	36.91	0.75
DXT1	MOL007923	2-(4-Hydroxyphenyl) ethyl (E)-3-(4-hydroxyphenyl) prop-2-enoate	93.36	0.21
HQ1	MOL000387	Bifendate	31.1	0.67
HQ2	MOL000033	(3S,8S,9S,10R,13R,14S,17R)-10,13-dimethyl-17-[(2R,5S)-5-propan-2-yloctan-2-yl]-2,3,4,7,8,9,11,12,14,15,16,17-dodecahydro-1h-cyclopenta[a]phenanthren-3-ol	36.23	0.78
HQ3	MOL000379	9,10-Dimethoxypterocarpan-3-O-*β*-D-glucoside	36.74	0.92
HQ4	MOL000296	Hederagenin	36.91	0.75
HQ5	MOL000442	1,7-Dihydroxy-3,9-dimethoxy pterocarpene	39.05	0.48
HQ6	MOL000422	Kaempferol	41.88	0.24
HQ7	MOL000098	Quercetin	46.43	0.28
HQ8	MOL000417	Calycosin	47.75	0.24
HQ9	MOL000439	Isomucronulatol-7,2′-di-O-glucosiole	49.28	0.62
HQ10	MOL000354	Isorhamnetin	49.6	0.31
HQ11	MOL000239	Jaranol	50.83	0.29
HQ12	MOL000371	3,9-di-O-methylnissolin	53.74	0.48
HQ13	MOL000211	Mairin	55.38	0.78
HQ14	MOL000380	(6aR,11aR)-9,10-dimethoxy-6a,11a-dihydro-6h-benzofurano[3,2-c] chromen-3-ol	64.26	0.42
HQ15	MOL000433	FA	68.96	0.71
HQ16	MOL000392	Formononetin	69.67	0.21
HQ17	MOL000378	7-O-methylisomucronulatol	74.69	0.3
GZ1	MOL000073	Ent-epicatechin	48.96	0.24
GZ2	MOL000492	(+)-catechin	54.83	0.24
GZ3	MOL001736	(−)-Taxifolin	60.51	0.27
GZ4	MOL004576	Taxifolin	57.84	0.27
DL1		Xanthine	GI absorption: High	
DL2		Guanidine	GI absorption: High	
DL3		Xanthinin	GI absorption: High	
DL4		4-Guanidino-1-butanol	GI absorption: High	
SZ		Crocetin	GI absorption: High	

**Table 4:** Top 11 related pathways in metascape for the ICH treatment of ZL capsule via ferroptosis.

GO	Description	Count	%	Log10 (*P*)	Log10 (*q*)	Hits
hsa05200	Pathways in cancer	17	51.52	−20.99	−18.57	CASP8, NQO1, EGFR, GSK3B, GSTP1, HMOX1, JUN, MYC, NFE2L2, MAPK1, PTEN, PTGS2, RB1, RELA, TGFB1, TGFB2, TP53
hsa05161	Hepatitis B	10	30.3	−14.91	−12.85	CASP8, JUN, MYC, MAPK1, RB1, RELA, TGFB1, TGFB2, TNF, TP53
hsa05163	Human cytomegalovirus infection	10	30.3	−13.47	−11.63	CASP8, EGFR, GSK3B, MYC, MAPK1, PTGS2, RB1, RELA, TNF, TP53
hsa04657	IL-17 signaling pathway	8	24.24	−13.07	−11.44	CASP8, GSK3B, JUN, MAPK1, PTGS2, RELA, TNF, TNFAIP3
hsa05418	Fluid shear stress and atherosclerosis	8	24.24	−11.69	−10.39	NQO1, GSTP1, HMOX1, JUN, NFE2L2, RELA, TNF, TP53
hsa05208	Chemical carcinogenesis - reactive oxygen species	8	24.24	−10.04	−8.9	NQO1, EGFR, HMOX1, JUN, NFE2L2, MAPK1, PTEN, RELA
hsa04216	Ferroptosis	5	15.15	−9.08	−7.99	ALOX15, ACSL4, HMOX1, SLC3A2, TP53
hsa01524	Platinum drug resistance	4	12.12	−5.91	−5.22	CASP8, GSTP1, MAPK1, TP53
hsa05012	Parkinson disease	5	15.15	−5	−4.39	HSPA5, NFE2L2, SNCA, TP53, UCHL1
hsa04217	Necroptosis	4	12.12	−4.57	−3.98	ALOX15, CASP8, TNF, TNFAIP3
hsa04370	VEGF signaling pathway	3	9.09	−4.43	−3.86	HSPB1, MAPK1, PTGS2

**Table 5:** Top 6 active ingredients of ZL capsule in above related 11 pathways.

ID	MolID	Compound	Degree	BetweennessCentrality	ClosenessCentrality
HQ7	MOL000098	Quercetin	18	0.23778696	0.51239669
SZ		Crocetin	6	0.08568377	0.41059603
HQ6	MOL000422	Kaempferol	6	0.01941172	0.41059603
A	MOL000358	Beta-sitosterol	4	0.01428604	0.40522876
HQ16	MOL000392	Formononetin	3	0.00604758	0.38509317
HQ10	MOL000354	Isorhamnetin	3	0.00570997	0.38509317

**Table 6:** Top 7 targets of ZL capsule in above 11 pathways.

Targets	Degree	BetweennessCentrality	ClosenessCentrality
PTGS2	24	0.44995211	0.55357143
RELA	10	0.04458046	0.41891892
JUN	9	0.03443671	0.41333333
TP53	8	0.068708	0.43055556
TNF	8	0.04903199	0.42465753
CASP8	8	0.03937065	0.41333333
GSK3B	8	0.05341178	0.38271605

## Data Availability

The data that support the findings of this study are available from the first author upon request.

## Supplementary Materials

Supplementary Materials The supplemental file of network pharmacology-related data in the article.
